# Glycyrrhizin protects mice against renal ischemia-reperfusion injury through inhibition of apoptosis and inflammation by downregulating p38 mitogen-activated protein kinase signaling

This article has been retracted.

**DOI:** 10.3892/etm.2014.1570

**Published:** 2014-02-21

**Authors:** SHAOJUN YE, YI ZHU, YINGZI MING, XINGGUO SHE, HONG LIU, QIFA YE

**Affiliations:** Research Center of the Chinese Health Ministry on Transplantation Medicine Engineering and Technology, The Third Xiangya Hospital, Central South University, Changsha, Hunan 410013, P.R. China

**Keywords:** glycyrrhizin, ischemia-reperfusion, kidney, inflammation, apoptosis

## Abstract

Ischemia-reperfusion (I/R) often leads to acute kidney injury, chronic renal failure and kidney transplantation failure. Glycyrrhizin is extracted from *Glycyrrhiza glabra* roots and is the predominant active component, which exhibits anti-inflammatory effects. However, to the best of our knowledge, the effect of glycyrrhizin on I/R-induced renal injury has not been investigated. In the present study, glycyrrhizin was demonstrated to attenuate renal I/R injury in mice via administration of glycyrrhizin, which suppressed the serum levels of creatinine and blood urea nitrogen 6 h following reperfusion; furthermore, the superoxide anions as well as the activity of superoxide dismutase within renal tissues was reduced by glycyrrhizin pretreatment. Moreover, the protein level of cleaved caspase-3, as well as its activity in renal tissue, was suppressed as a result of the glycyrrhizin pretreatment, indicating that glycyrrhizin inhibits I/R-induced renal cell apoptosis. In addition, glycyrrhizin pretreatment appeared to ameliorate I/R-induced renal injury via inhibition of inflammatory cell infiltration, as well as the production of pro-inflammatory cytokines, including tumor necrosis factor-α, interferon-γ, interleukin (IL)-1β and IL-6. The underlying molecular mechanism was investigated and it was shown that the activity of p38 mitogen-activated protein kinase signaling was downregulated as a result of glycyrrhizin administration. In conclusion, the present study indicated that glycyrrhizin provided significant protection against I/R-induced renal injury in mice by inhibiting inflammatory responses and renal cell apoptosis. Therefore, glycyrrhizin may be used in abdominal surgery and kidney transplantation for the prevention of renal I/R damage.

## Introduction

Ischemia-reperfusion (I/R)-induced kidney injury results from a sudden transient reduction in blood flow, arising from shock, trauma, abdominal surgery or kidney transplantation, and often leads to acute kidney injury, chronic renal failure or failure of the kidney transplant (1–3). Previous studies have identified that I/R leads to the activation and infiltration of neutrophils and macrophages, which release numerous pro-inflammatory mediators that trigger acute inflammatory responses; this has been demonstrated to be crucial in I/R-induced renal injury (4–7). In addition, renal cell apoptosis may be involved in I/R-induced renal injury.

Glycyrrhizin is the predominant active component that is extracted from the roots of *Glycyrrhiza glabra* and exhibits anti-inflammatory effects (8). Furthermore, glycyrrhizin has been reported to attenuate I/R-induced gut, spinal cord, liver and heart damage (9–14). However, to the best of our knowledge, the effect of glycyrrhizin on I/R-induced renal injury has not been investigated.

## Materials and methods

### Renal I/R procedure

The animal experiments in the present study were approved by the Ethics Committee of the Third Xiangya Hospital, Central South University (Changsha, China). Male C57BL/6 mice (age, 12 weeks; weight, 20–25 g) were housed at Xiangya Medical Experimental Animal Center, Central South University in a laminar flow, temperature-controlled, pathogen-free environment under a 12 h light/dark cycle. The mice were fasted for 24 h prior to the experiments and provided with tap water *ad libitum*. During surgery, an intraperitoneal injection of 50 mg/kg pentobarbital was administered to anesthetize the mice. Bilateral flank incisions were made, the right kidney was removed and the left kidney was subjected to ischemia using a microvascular clamp, which was removed after 30 min and the wound was closed. To induce ischemia of the left kidney, a microvascular clip was used to clamp the renal artery after a transverse incision was made to the abdomen. Half an hour later, the clamp was removed, and the wound was closed. The mice were divided into three groups of six; in the sham-operated group, the mice underwent anesthesia, bilateral flank incisions and a right nephrectomy. In the glycyrrhizin-treated group, the mice were injected with 60 mg/kg glycyrrhizin using an infusion pump (Chizhou Kangyuan Medical Equipment Co., Ltd. Chizhou, China) 1 h prior to ischemia. In the saline-treated group, the mice were administered with 60 mg/kg saline. The mice were sacrificed by cervical dislocation under anesthesia 6 h after reperfusion and the blood and kidney samples were immediately collected.

### Assessment of kidney function

Renal function was assessed via observation of serum creatinine (Cr) and blood urea nitrogen (BUN) levels at the Clinical Laboratory of the Third Xiangya Hospital, Central South University (Changsha, China).

### Assessment of the renal tissue superoxide anion (SOA) level

An SOA assay kit (Sigma, St. Louis, MO, USA) was used to determine the level of SOA in the soluble fraction of renal tissue in accordance with the manufacturer’s instructions and the reaction was analyzed using a spectrophotometer (Shimadzu, Kyoto, Japan) at a wavelength of 550 nm.

### Assessment of the renal tissue superoxide dismutase (SOD) activity

The SOD activity was measured using the SOD activity assay kit (Biovision, Milpitas, CA, USA) based on the inhibition of adenochrome production by SOD during epinephrine auto-oxidation. Changes in fluorescence were read at a wavelength of 480 nm (Microplate Reader; Bio-Rad, Hercules, CA, USA).

### Caspase-3 activity measurement

Caspase-3 colorimetric assay kit (Biovision, San Francisco Bay Area, CA, USA) was used to determine the activity of caspase-3, according to the manufacturer’s instructions. Briefly, 20 μg kidney cytosolic protein was extracted and incubated in a solution buffer at room temperature for 30 min. The reaction was initiated by the addition of 200 μM N-acetyl-Asp-Glu-Val-Asp-7-amino-4-trifluoromethylcoumarin and incubated at 37°C for 2 h. The change in absorbance was measured spectrophotometrically at a wavelength of 400 nm.

### Myeloperoxidase (MPO) activity measurement

MPO is a neutrophil-specific enzyme, the presence of which is considered to be an indicator of neutrophil infiltration in the kidney. Renal tissues were homogenized on ice in phosphate-buffered saline (PBS) with 0.5% hexadecyltrimethyl ammonium bromide (Sigma) and 0.146% EDTA (pH 6.0). The homogenates were centrifuged at 13,400 × g for 30 min at 4°C and the supernatant was incubated at 60°C for 2 h. Hydrogen peroxide (0.005%) and 0.167 mg/ml O-dianisidine dihydrochloride (Sigma) in PBS (pH 6.0) was added and the change in absorbance was measured spectrophotometrically at a wavelength of 460 nm.

### Serum pro-inflammatory cytokine measurements

Enzyme-linked immunosorbent assay kits (mouse TNF-α ELISA kit, Mouse IFN-γ ELISA kit, mouse IL-1β ELISA kit, mouse IL-6 ELISA kit; Sigma) were used to determine the serum levels of the key pro-inflammatory cytokines, including tumor necrosis factor (TNF)-α, interferon (IFN)-γ, interleukin (IL)-1β and IL-6, in accordance with the manufacturer’s instructions.

### Western blot assay

Cytoplasmic extraction reagents (Pierce Biotechnology, Inc., Rockford, IL, USA) were used to extract the cytosolic proteins from the mice kidney tissues, in accordance with the manufacturer’s instructions. After determining the concentration of protein using the Enhanced BCA Protein Assay kit (Beyotime, Shanghai, China), 20 μg protein was separated using 10% SDS-PAGE, which was transferred to nitrocellulose membranes and maintained at room temperature for 1 h in a buffer solution containing 5% dried skimmed milk. The membrane was incubated at room temperature for 3 h with mouse anti-total-p38 MAPK, mouse anti-phospho-p38 MAPK, mouse anti-cleaved caspase-3 or mouse anti-GAPDH monoclonal antibodies (Abcam, Cambridge, UK), and subsequently with goat anti-mouse secondary antibody (Abcam) for 1 h. The signals on the membranes were detected using an enhanced chemiluminescence reagent (PerkinElmer, Waltham, MA, USA) and the densitometry was analyzed by Image-Pro plus software 6.0 (Media Cybernetics, Inc., Rockville, MD, USA).

### Statistical analysis

All of the data were expressed as means ± standard deviation and analyzed by one-way analysis of variance, followed by Student’s t-test to assess the statistical significance. P<0.05 was considered to indicate a statistically significant difference.

## Results

### Administration of glycyrrhizin protects mice from I/R-induced renal injury

To investigate the effect of glycyrrhizin on I/R-induced renal injury in mice, the serum levels of Cr and BUN were examined 6 h following reperfusion. The mice in the saline-treated group showed significantly higher serum levels of Cr and BUN compared with the mice in the sham-operated group, which indicated marked I/R-induced renal damage. However, the mice that were administered with glycyrrhizin exhibited notably lower serum levels of Cr and BUN, when compared with those in the saline-treated group. These findings indicate that pretreatment with glycyrrhizin provides effective protection against I/R-induced renal injury in mice (Fig. 1A and B).

The SOA level that was observed in the soluble fraction of the renal tissue 6 h after reperfusion was significantly higher in the saline-treated control group, when compared with that observed in the sham-operated and glycyrrhizin-treated groups (Fig. 1C). In addition, the SOD activity in the kidney tissue following I/R was examined and it was demonstrated that the SOD activity was greater in the glycyrrhizin-treated group than in the saline-treated group (Fig. 1D).

### Administration of glycyrrhizin attenuates I/R-induced renal cell apoptosis in mice

To further investigate the effect of renal cell apoptosis in I/R-induced renal injury, western blot analysis was performed to determine the expression of cleaved caspase-3, 6 h after reperfusion. The expression level was notably reduced in the mice that were pretreated with glycyrrhizin when compared with that of the mice pretreated with saline. For further confirmation, the activity of caspase-3 in the renal tissues was determined in each group (Fig. 2A). Consistently, the activity of caspase-3 was downregulated in the mice from the glycyrrhizin-treated group compared with the saline-treated group. Therefore, it was hypothesized that glycyrrhizin protects against I/R-induced renal damage in mice, partially via the inhibition of renal cell apoptosis.

### Administration of glycyrrhizin attenuates I/R-induced renal inflammation in mice

As neutrophil and macrophage infiltration is key in I/R-induced tissue inflammation, and MPO activity is a key indicator of neutrophil and macrophage infiltration, the MPO activity in the renal tissue of each group was assessed. The activity of MPO was identified to be significantly upregulated in the saline-treated group compared with the sham-operated group. However, the activity of MPO in the glycyrrhizin-treated group was significantly reduced compared with the saline-treated group with a value that was comparable to the sham-operated group (Fig. 3A).

To identify the mechanism involved, the effect of glycyrrhizin on the production of inflammatory cytokines, including TNF-α, IFN-γ, IL-1β and IL-6 was examined; these inflammatory cytokines have been demonstrated to be significant in the induction of renal I/R injury (15,16). The production of pro-inflammatory TNF-α, IFN-γ, IL-1β and IL-6 was significantly reduced in the glycyrrhizin-treated mice, when compared with that observed in the saline-treated mice 6 h after reperfusion (Fig. 3B). Accordingly, these findings indicate that pretreatment with glycyrrhizin ameliorates I/R-induced renal injury via the mediation of inflammatory cell infiltration in addition to the production of inflammatory cytokines.

### Administration of glycyrrhizin suppresses p38 MAPK activation during I/R

As glycyrrhizin has been reported to exhibit a suppressive effect on the activation of the p38 MAPK pathway in I/R-induced myocardial injury in rabbits, it was hypothesized that it may be similarly involved in the regulation of the p38 MAPK pathway in renal I/R damage in mice. Thus, the activity of the p38 MAPK pathway in the renal tissues was determined in each group via western blot assay. The phosphorylated-p38 MAPK protein level in the saline-treated group was significantly increased compared with the sham-operated group; however, the phosphorylated-p38 protein level in the glycyrrhizin-treated group was notably reduced compared with that in the saline-treated group (Fig. 4). These findings confirmed the hypothesis that administration of glycyrrhizin suppressed the activation of p38 MAPK in I/R-induced renal damage in mice.

## Discussion

Glycyrrhizin has been identified to exhibit a protective effect on I/R-induced organ damage, including damage to the gut, liver and heart (9–13). However, whether glycyrrhizin protects against I/R-induced renal injury has not previously been analyzed. In the present study, the effect of glycyrrhizin on I/R-induced kidney injury in mice was investigated. To the best of our knowledge, this is the first study to show that pretreatment with glycyrrhizin attenuates renal I/R injury via inhibition of tissue inflammation as well as protection against cell apoptosis, indicating that glycyrrhizin may be used for the prevention of I/R-induced kidney injury in clinical settings.

Renal cell apoptosis has been shown to be key in I/R-induced renal damage (17). Among the apoptotic mediators, activated caspase-3 acts as a final executor, as it regulates the extrinsic and intrinsic pathways of apoptosis (18,19). Furthermore, caspase-3-mediated cell apoptosis has been demonstrated to be essential in I/R-induced organ damage (20); thus, the effect of glycyrrhizin on I/R-induced renal cell apoptosis was investigated in the present study. The findings showed that administration of glycyrrhizin notably inhibited the protein level of cleaved caspase-3, (the activated form of caspase-3) within the renal tissues. Moreover, the activity of caspase-3 was downregulated as a result of glycyrrhizin administration. Therefore, it is hypothesized that glycyrrhizin may protect renal cells against I/R-induced apoptosis by suppressing caspase-3.

Tissue I/R damage has been identified to predominantly result from I/R-induced excessive inflammatory responses (21). When renal I/R occurs, neutrophils and macrophages initially infiltrate into the damaged kidney and secrete large quantities of pro-inflammatory mediators, which promote the infiltration of neutrophils and macrophages into the damaged tissues and further promote tissue inflammatory responses (22,23). Furthermore, infiltrated neutrophils and macrophages reduce renal blood flow, which leads to microcirculatory failure (24,25). To investigate the effect of glycyrrhizin on I/R-induced neutrophil and macrophage infiltration into damaged renal tissues, the activity of MPO, an enzyme specific to neutrophils and macrophages, was examined. The findings indicated that the administration of glycyrrhizin protects against I/R-induced macrophage and neutrophil infiltration in the renal tissue of mice. Consistently, the following findings demonstrated that the secretion of pro-inflammatory cytokines, including TNF-α, IFN-γ, IL-1β and IL-6, was markedly lower in the glycyrrhizin-treated mice compared with the saline-treated mice. Similarly, the production of IL-10, a key anti-inflammatory cytokine, was significantly higher in glycyrrhizin-treated mice compared with saline-treated mice. In addition, glycyrrhizin has been demonstrated to protect against I/R-induced tissue damage by suppressing the inflammatory response. Liu *et al* (11) identified that administration of glycyrrhizin reduced the serum levels of pro-inflammatory cytokines, including TNF-α, IL-6 and IL-8, in I/R-induced myocardial injury in rabbits. Zhai *et al* (13) indicated that the administration of glycyrrhizin significantly decreased the levels of serum TNF-α and IL-6, which protected the rat hearts against I/R injury. In accordance with these previous findings, the data from the present study indicated that glycyrrhizin protects mice against I/R-induced renal injury, via the inhibition of inflammatory responses.

The activation of p38 MAPK signaling is known to be significant in I/R-induced cell apoptosis as well as in inflammatory responses (26,27); for example, administration of C-phycocyanin protected against I/R-induced cardiomyocyte apoptosis in rats by inhibiting I/R-induced p38 activation (28). Furthermore, it has been reported that glycyrrhizin attenuated I/R-induced myocardial damage in rabbits by suppressing the production of certain inflammatory cytokines through the p38 MAPK pathway (11). Thus, it was hypothesized in the present study that the protective function of glycyrrhizin against I/R-induced renal cell apoptosis and inflammatory responses may occur through inhibition of p38 MAPK activation. The results of the western blot analysis conducted in the present study showed that glycyrrhizin significantly suppressed the phosphorylated-p38 protein level, demonstrating that glycyrrhizin attenuated the I/R-induced activation of p38 MAPK signaling, which resulted in a protective effect against renal cell apoptosis and inflammatory responses in I/R-induced kidney injury in mice.

In conclusion, the present study demonstrated that pretreatment with glycyrrhizin provided marked protection for mice against I/R-induced renal injury via inhibition of inflammatory responses and renal cell apoptosis. Therefore, the administration of glycyrrhizin may be effective in the prevention of I/R-induced renal injury in abdominal surgery and kidney transplantation.

## Figures and Tables

**Figure 1:** (A) Serum Cr level, (B) BUN level and renal tissue (C) SOA level and (D) SOD activity was examined in each group. ^**^P<0.01. CR, creatinine; I/R ischemia-reperfusion; Gl, glycyrrhizin; SOA, superoxide anions; SOD, superoxide dismutase.

**Figure 2:** (A) Western blot analysis was performed to examine the protein level of cleaved caspase-3 in the three groups. GAPDH served as an internal control. (B) Activity of caspase-3 in the renal tissue was determined in each group using a caspase-3 colorimetric assay kit. ^*^P<0.05 and ^**^P<0.01. I/R, ischemia-reperfusion; Gl, glycyrrhizin.

**Figure 3:** (A) Activity of MPO in the renal tissue was determined in the three groups. (B) The serum levels of key pro-inflammatory cytokines, including TNF-α, IFN-γ, IL-1β and IL-6, were examined in each group using enzyme-linked immunosorbent assay kits. ^*^P<0.05 and ^**^P<0.01. MPO, myeloperoxidase; I/R, ischemia-reperfusion; Gl, glycyrrhizin; TNF, tumor necrosis factor; IFN, interferon; IL, interleukin.

**Figure 4:** Protein levels of phosphorylated-p38 MAPK and total-p38 MAPK in the renal tissue were examined in the three groups using western blot analysis. GAPDH served as an internal control. ^*^P<0.05 and ^**^P<0.01. I/R, ischemia-reperfusion; Gl, glycyrrhizin; MAPK, mitogen-activated protein kinase.
